The article "Statins significantly repress rotavirus replication through downregulation of cholesterol synthesis" was retracted in 2022. Reasons: no approval from the institution; concerns about the authorship.

# Statins significantly repress rotavirus replication through downregulation of cholesterol synthesis

**DOI:** 10.1080/19490976.2021.1955643

**Published:** 2021-08-07

**Authors:** Shihao Ding, Bingting Yu, Anneke J. van Vuuren

**Affiliations:** a Department Of Gastroenterology And Hepatology, Na-1001, Erasmus MC – University Medical Center Rotterdam, CA Rotterdam, Netherlands; b Department of Endocrinology and Metabolism, Amsterdam University Medical Center, University of Amsterdam, Amsterdam, Netherlands; c Netherlands Institute for Neuroscience, Royal Netherlands Academy of Arts and Sciences, Amsterdam, Netherlands

**Keywords:** Rotavirus infection, cholesterol synthesis, statins, antiviral therapy

## Abstract

Rotavirus is the most common cause of severe diarrhea among infants and young children and is responsible for more than 200,000 pediatric deaths *per* year. There is currently no pharmacological treatment for rotavirus infection in clinical activity. Although cholesterol synthesis has been proven to play a key role in the infections of multiple viruses, little is known about the relationship between cholesterol biosynthesis and rotavirus replication. The models of rotavirus infected two cell lines and a human small intestinal organoid were used. We investigated the effects of cholesterol biosynthesis, including inhibition, enhancement, and their combinations on rotavirus replication on these models. The knockdown of 3-hydroxy-3-methylglutaryl-CoA reductase (HMGCR) was built by small hairpin RNAs in Caco2 cells. In all these models, inhibition of cholesterol synthesis by statins or HMGCR knockdown had a significant inhibitory effect on rotavirus replication. The result was further confirmed by the other inhibitors: 6-fluoromevalonate, Zaragozic acid A and U18666A, in the cholesterol biosynthesis pathway. Conversely, enhancement of cholesterol production increased rotavirus replication, suggesting that cholesterol homeostasis is relevant for rotavirus replication. The effects of all these compounds toward rotavirus were further confirmed with a clinical rotavirus isolate. We concluded that rotavirus replication is dependent on cholesterol biosynthesis. To be specific, inhibition of cholesterol synthesis can downregulate rotavirus replication; on the contrary, rotavirus replication is upregulated. Statin treatment is potentially an effective novel clinical anti-rotavirus strategy.

## Introduction

Rotavirus is a non-enveloped double-stranded RNA (dsRNA) virus that has a complex architecture of three concentric capsid layers that surround a genome of 11 segments of dsRNA, the viral RNA-dependent RNA polymerase and the viral-capping enzyme. Rotavirus is ubiquitous globally and infects virtually every child of <2 y of age.^1,2^ The estimate for the associated global mortality reaches over 200,000 casualties *per anum.^3^* Although vaccination is an effective approach to prevent rotavirus infection, the virus-induced diarrhea is still a heavy burden worldwide, as the most terrible cases occur in developing countries where access to rotavirus vaccination is limited and where the licensed rotavirus vaccines are less efficacious and efficient than in high-income countries.^4,5^ Oral or intravenous rehydration remains currently the mainstream treatment for rotavirus infection, but it is passive and cannot shorten the diarrhea duration.^6^ Evidence for the potential efficacy of conventional antivirus drugs to rotavirus has been provided, but their uses are commonly hampered due to the side effects and the economic considerations.^2^ Obviously, the improvement of the treatment strategy for rotavirus infection is urgent. A better understanding of the physiological mechanism of rotavirus infection may provide an important insight leading to an improvement for rotavirus infection therapeutics.

The article "Statins significantly repress rotavirus replication through downregulation of cholesterol synthesis" was retracted in 2022. Reasons: no approval from the institution; concerns about the authorship.

Rotavirus primarily infects and replicates in the villi and enteroendocrine cells of host small intestine.^7^ Cholesterol plays an important role in both intestinal physiology and anti-virus responses.^8–10^ Specific to rotavirus, the presence of cholesterol on the plasma membrane is an important prerequisite in the process of rotavirus infection.^11^ The interaction between rotavirus VP4 protein with lipid-raft, which is described as the rich cholesterol micro-domains on cell membrane, promotes the assembly of rotavirus.^12^ Treating with Methyl-beta-cyclodextrin (MβCD) which is known to extract cholesterol from cell membrane can prevent rotavirus infection.^13^ Although the evidence that cholesterol on cell membrane is essential for rotavirus infection has been provided, the importance of cholesterol metabolism for rotavirus replication remains largely obscure.

Intracellular cholesterol synthesis is mainly dependent on the mevalonate pathway, and HMGCR is the rate-controlling enzyme of the cholesterol synthesis pathway.^14^ Pharmacologically, as the competitive inhibitor of HMGCR, statin inhibits the HMGCR-dependent cholesterol biosynthesis.^15^ Statin is one of the globally best-selling drugs to reduce the morbidity and mortality in patients with hypercholesterolemia.^16^ Importantly, statin is generally considered to be safe after decades of prolonged use for adults and even children.^17,18^ Also in the context of intestinal physiology, the benefit profile of statin is very marked. Statin contributes to the regeneration of intestine epithelia, which is an important consideration when taking the epithelial damage caused by rotavirus infection into account.^19^ If rotavirus replication interacts with cholesterol synthesis, it could provide a new strategy to against rotavirus infection in clinical work.

The article "Statins significantly repress rotavirus replication through downregulation of cholesterol synthesis" was retracted in 2022. Reasons: no approval from the institution; concerns about the authorship.

Herein, we evaluated the anti-rotavirus potentials of three different statins: atorvastatin, lovastatin, and simvastatin toward two different rotavirus isolates: simian rotavirus SA11 strain and human rotavirus 026 K strain. We observed the potent anti-rotavirus functions of all the statins in Caco2 and MA104 cells and primary HSI organoids, and the inhibitory effects were dose- and time-dependent. These statins also drastically reduced the number of produced progeny rotavirus particles, suggesting statin could impair the spread of rotavirus. The similarly inhibitory results were also observed by the other inhibitors in the cholesterol synthesis pathway. Conversely, enhancing cholesterol production could apparently upregulate rotavirus replication. The valuable results unveiled that rotavirus replication has a close relationship with HMGCR-dependent cholesterol synthesis, and it also provided an important reference for using statin to treat rotavirus infection.

## Materials and methods

### Reagents, antibodies, and plasmids

Atorvastatin, Lovastatin, Simvastatin, 6-fluoromevalonate, Zaragozic acid A (ZA-A), U18666A, R-mevalonate acid (R-MA0 and Cholesterol were purchased from Sigma-Aldrich (St Louis, MO, USA). All the reagents were dissolved in Dimethylsulfoxide (DMSO). The mouse monoclonal antibody against rotavirus VP4 protein was a gift from Prof. Harry Greenberg (Medicine-Gastroenterology & Hepatology, School of Medicine, Stanford University, USA). The mouse antibody against the rotavirus VP6 protein and the antibody against HMGCR were purchased from Abcam (Cambridge, MA, USA). The mouse antibody against β-actin was obtained from Santa Cruz Biotechnology (Dallas, TX, USA). The secondary antibodies were obtained from Dako (for western blotting; Amstelveen, the Netherlands) and Invitrogen (for immunofluorescence; Carlsbad, CA, USA) respectively. HMGCR knockdown small hairpin RNA (shRNA) were purchased from Erasmus MC biobank and described in supplement table 1.

### Cells, HSI organoids, and rotavirus strains

Human epithelial colorectal adenocarcinoma cell line Caco2, human embryonic kidney epithelial cell line 293 T (HEK 293 T) and African green monkey fetal kidney cell line MA104 were originally purchased from ATCC (Manassas, VA, USA). Caco2 cells and MA104 cells were maintained in Dulbecco’s modified eagle medium (DMEM) (Lonza, Verviers, Belgium) supplemented with 20% and 10% (v/v) heat-inactivated Fetal calf serum (FCS; Sigma–Aldrich, St. Louis, MO, USA), respectively, with 100 U/mL Penicillin/Streptomycin (P/S; Gibco, Grand Island, USA) solution. HEK 293 T cells were cultured with the same medium of MA104 cells. All the cells were incubated at 37°C with 5% CO_2_. The cells were analyzed by genotyping to confirm mycoplasma negative.

The article "Statins significantly repress rotavirus replication through downregulation of cholesterol synthesis" was retracted in 2022. Reasons: no approval from the institution; concerns about the authorship.

Human intestinal tissues were surgically resected and transferred into a 15 mL falcon tube including 10 mL Complete chelating solution (CCS; Milli-Q H_2_O was supplemented with 1.0 g/L Na_2_HPO_4_-2H_2_O, 5.6 g/L NaCl, 1.08 g/L KH_2_PO_4_, 15 g/L Sucrose, 0.12 g/L KCl, 10 g/L D-Sorbitol and 80 µg/L DL-dithiothreitol). The study was approved by the ethics committee of Erasmus University Medical Center in Rotterdam.

Simian rotavirus SA11 strain was a kind gift from Karen Knipping (Nutricia Research Utrecht, the Netherlands). Patient-derived rotavirus strain, 026 K, was isolated from the stool sample that was taken during the patient diarrhea period and stored in Erasmus MC biobank.

## Rotavirus infection and pharmacological treatments

Caco2 and MA104 cells were expanded and subjected to rotavirus infection as described earlier.^20^ The rotavirus infection process of human small intestinal (HIS) organoids has been extensively described before.^21,22^

Specific drug was added with corresponding concentrations post-rotavirus infection. Refresh the culture medium with the drug every 24 hours. After 48 hours incubation, the infected cells were collected for subsequent experiments.

### RNA extraction and quantitative real-time polymerase chain reaction (qRT-PCR) analysis

The intracellular RNA was isolated using a Nucleo Spin® RNA kit (MACHEREY-NAGEL, Düren, Germany) and quantiﬁed with a Nanodrop ND-1000 (Wilmington, DE, USA). cDNA was transcribed with 0.5 mg the RNA, and was diluted 1:10. Two μL the cDNA was used for qRT-PCR with the primers (as described in supplementary table 2). For the extraction of the extracellular rotavirus RNA, the supernatant of the cells was collected for lysis using the same Nucleo Spin® RNA kit according to the manufacturers’ instructions. The process of extracellular RNA extraction was equal to that in the intracellular RNA isolation.

All qRT-PCR experiments were performed with SYBR Green-based real-time PCR and the Step One Plus System (Thermo Fisher Scientiﬁc Life Sciences; Carlsbad, CA, USA). The relative expressions of target messenger RNA (mRNAs) were normalized to Glyceraldehyde 3-phosphate dehydrogenase (GAPDH). The analysis of gene expression was calculated by the comparative threshold cycle measurement.^21,23^

### Rotavirus RNA copies assay by long-term

qRT-PCR was used for measuring the intracellular rotavirus RNA copies of Caco2 cells by long-term. After rotavirus SA11 infection, Caco2 cells were collected immediately, followed by RNA isolation and the measurement of the rotavirus RNA genome by qRT-PCR. During the next 96 hours, every 24 hours the intracellular rotavirus RNA copies were assayed as before and compared to the original expression of the control or the drug treatment, respectively.

The article "Statins significantly repress rotavirus replication through downregulation of cholesterol synthesis" was retracted in 2022. Reasons: no approval from the institution; concerns about the authorship.

### Western blotting

Western blotting process was described as previously.^21^ Proteins were detected and quantified by a LI-COR Odyssey infrared scanner (LI-COR Bioscience; Lincoln, NE, USA). The scanned data was analyzed using an Odyssey version 3.0 software (LI-COR Bioscience; Lincoln, NE, USA).

### Immunofluorescence (IF) staining

IF staining was performed as described previously.^20^ The imaging of Caco2 and MA104 cells was performed by the Olympus IX70 fluorescence microscope.

IF staining process of HSI organoids was similar to the cellular staining process. The imaging was performed by the Leica TCS LSI confocal microscope.

### Lentivirus-mediated RNA interference

All shRNA HMGCR vectors were purchased from Erasmus MC Biobank. The production process of the target lentivirus plasmids was similar as described before.^24^ To generate the stable HMGCR knockdown cell line, Caco2 cells were inoculated with the vectors of lentivirus plasmids for 6 hours. Afterward, the cells were selected with 8 μg/mL puromycin (Sigma–Aldrich; St. Louis, MO, USA) in DMEM medium with 20% (v/v) FCS for more than 7 days. After confirming the HMGCR knockdown effects by qRT-PCR and western blotting, the optimal HMGCR knockdown Caco2 cells with two distinct shRNA vectors were selected for further experiments.

### Cell viability and 50% maximal inhibitory concentration (IC_50_) calculation

The viabilities of Caco2 and MA104 cells with all the compounds treatments were determined by 3-(4, 5Dimethylthiazol-2-yl)-2,5-diphenyl-tetrazolium bromide (MTT; Invitrogen; Carlsbad, CA, USA) assay. Around 5 × 10^4^ Caco2 or MA104 cells were seeded into each well of 96-well plate with 3 repeated wells to incubate with the specific compound concentration. These cells were refreshed by the medium every 24 hours. After 48 hours, followed by adding 10 µL of 500 μg/mL MTT solution to each well and incubated at 37°C for 3 hours. Subsequently, the medium was removed and replaced with 100 μL DMSO to incubate at 37°C for 30 min. Testing was performed by a Perseptive biosystems 4000 multi-well plate reader (CYTOFLUOR; USA).

Based on the results of three independent MTT assay, the IC_50_ value was calculated. A four parameters logistic regression model was used for the calculation: Y = Min + ((Max – Min)/1 + (X/C50) Hill coefficient) using online IC_50_ calculator of AAT Bioquest at https://www.aatbio.com/tools/ic50-calculator.

The article "Statins significantly repress rotavirus replication through downregulation of cholesterol synthesis" was retracted in 2022. Reasons: no approval from the institution; concerns about the authorship.

### Virus titer assay

The original supernatant was serially diluted 11 times from 10^−1^ to 10^−11^ to measure 50% tissue culture infectious doses (TCID_50_). Briefly, each dilution was inoculated into the monolayer confluent MA104 cells in a well of 96-well plate with eight repeated wells under 37°C for 1 h. After the incubation, the monolayer cells were washed by PBS, and cultured with DMEM to incubate at 37°C for 72 h. The Log_10_ TCID_50_ was calculated using the Reed–Muench method as described previously.^25^

### Statistical analysis

Statistical analysis was performed by the non-paired, non-parametric test (Mann–Whitney test; GraphPad Software, San Diego, CA, USA). Statistical significance was defined as *P < .05, **P < .005, ***P < .001.

## Results

### Statins significantly repressed rotavirus replication

Given rotavirus primarily infects the small intestinal epithelial cells of host, Caco2 cells should be an ideal cell model for studying the virus infection.^26^ Because of the heterogeneities of molecular structure, efficacy and pharmacokinetics across distinct statins.^27^ To avoid the potential statin-dependently specificity, we chose three different statins for our investigation. As evident from Figure 1a, the notable and dose-dependent decreases of the rotavirus RNA copies were observed, which dropped to 7%, 20%, and 16% intracellularly at 50 µM of atorvastatin, lovastatin, and simvastatin, respectively; correspondingly, decreased to 3%, 8%, and 7% extracellularly. By the three statins treatments, and the expressions of the rotavirus structural VP4 and VP6 proteins were also repressed evidently (Figure 1b, Figure S1a; Figure 2b). The data indicated that statin significantly inhibited rotavirus replication in Caco2 cells. To avoid the potential issue relating to the cellular specificity, we proceeded to investigate the effects of the statins in MA104 cell line which was previously reported to support favorably the infection and replication of rotavirus.^28^ In MA104 cells, the results were essentially identical to these in Caco2 cells (Figure 1c and d, Figure S1b and 2 c). In parallel, the viabilities of Caco2 and MA104 cells were not markedly affected by the tested statins concentrations using IC_50_ assay (Figure S1d and e). To better characterize the anti-rotavirus effect of statin under physiological conditions, we performed the confirmatory experiment with HSI organoids that included the characteristics of the intestinal epithelia, as well as the existence of the villus domain and crypt domain.^29^ Consistently, all the statins significantly blocked rotavirus replications (Figure 1e and f, and Figure S1c). All the results concluded that statin could effectively repress rotavirus replication.

The article "Statins significantly repress rotavirus replication through downregulation of cholesterol synthesis" was retracted in 2022. Reasons: no approval from the institution; concerns about the authorship.

**Figure 1.** Statins impair rotavirus replication. (a) Caco2 cells were infected with rotavirus SA11 strain (MOI 0.7) and subsequently treated with different concentrations of atorvastatin (n = 7), lovastatin (n = 7), or simvastatin (n = 5) for 48 hours, then the intra- (left) and extracellular (right) rotavirus RNA levels were measured by qRT-PCR, and (b) rotavirus VP4 protein were measured with 50 µM atorvastatin, lovastatin, and simvastatin treatment for 48 hours respectively by western blot. In MA104 cells, (c) treated as described in a, the intra- (left) and extracellular (right) rotavirus RNA levels with the three statins treatments respectively (n = 5), and (d) the expressions of the rotavirus VP4 protein, treated as described in b. In HSI organoids, (e) treated as described in a, the inner rotavirus RNA level with the treatments of the three statins respectively (n = 3), and (f) the expression of rotavirus VP4 protein, treated as described in b. (g) The titers of infectious rotavirus particles were measured by TCID_50_ assays with 50 µM three statins treatments respectively in MA104 cells (n = 6). (h) The 96-hour time course experiments of atorvastatin (left), lovastatin (middle), and simvastatin (right) treatments respectively (n = 3) on the intracellular rotavirus RNA replication. All data presented as mean ± SEM, *p < .05, **p < .01, ***p < .001

**Figure 2.** **Statins inhibit the expressions of rotavirus VP6 protein**. (a) Schematic depiction of the inhibitors of cholesterol biosynthesis. Following the infection of rotavirus SA11 strain (MOI 0.7) with 50 µM atorvastatin, lovastatin, or simvastatin treatment for 48 hours respectively, the expression of rotavirus VP6 protein was observed by IF staining in Caco2 cells (b), MA104 cells (c) and HSI organoids (d). VP6 protein was green, and the nuclei of the cells were visualized by DAPI (blue). The results showed that statins significantly reduced the expression of rotavirus VP6 protein

Additionally, to clarify the effect of statin on the infectious rotavirus particles, the titer of rotavirus in supernatant was measured by TCID_50_ assay. As shown in Figure 1g, the titer of rotavirus with the statins treatments distinctly dropped compared to the control. To track the anti-rotavirus effect of statin by time, we performed the 96-h time course experiments for all the statins on the intracellular rotavirus RNA level by qRT-PCR. The virus RNA levels declined since the first 24 hours and maintained at a relatively low standard during the whole course, revealing the anti-rotavirus effect of statin was time-dependent (Figure 1h).

The article "Statins significantly repress rotavirus replication through downregulation of cholesterol synthesis" was retracted in 2022. Reasons: no approval from the institution; concerns about the authorship.

### Rotavirus replication required HMGCR-dependent pathway

The anti-rotavirus function of statin could be explained that rotavirus replication required HMGCR-dependent activity. Pharmacological inhibitor, however, could have the off-target effect that created the biological activities. Also for statin, relevant HMGCR-independent activities had been described.^30^ Therefore, to address the potential issue, we decided to investigate the effect of HMGCR on rotavirus replication in Caco2 cells. Following the primary investigation of a panel of shRNA HMGCR vectors in combination with lentivirus transduction on HMGCR expression by qRT-PCR (Figure 3a), as the two most effective vectors, sh10952 and sh10955 were selected to be further confirmed by western blotting analysis (Figure 3b). Subsequently, the transductions of a scrambled control vector and the shRNA HMGCR vectors were contrasted for their potentialities to support rotavirus. As the evidence from (Figure 3c,d) and e, the reduction of HMGCR markedly impaired rotavirus replication on both RNA and protein levels. According to the data, the HMGCR-dependent pathway was critical for rotavirus infection, confirming the anti-rotavirus effect of statin was related to its HMGCR inhibition.

**Figure 3.** **shRNA-mediated HMGCR knockdown in Caco2 cells represses rotavirus replication**. (a) Lentiviral shRNA vectors, targeting HMGCR gene or non-targeted control lentivirus were produced in HEK 293 T cells. Subsequently, the transductions of the lentiviral shRNA vectors were performed in Caco2 cells. qRT-PCR analysis was conducted to detect the RNA levels of HMGCR among shRNA 10951–10955 HMGCR vectors. (b) Based on the qRT-PCR analysis, the HMGCR knockdown effects of sh10952 and sh10955 vectors were confirmed by western blot analysis (n = 3). (c) The HMGCR knockdown significantly inhibited the intracellular rotavirus RNA replications post-infection 48 hours (n = 6), and (d) the decreased expressions of rotavirus VP4 protein by western blot analysis (n = 3). (e) The decreased expressions of rotavirus VP6 protein by HMGCR knockdown. VP6 protein was stained as green, and nuclei were visualized by DAPI (blue). All data presented as mean ± SEM, *p < .05, **p < .01, ***p < .001

### Inhibitions of cholesterol synthesis impaired rotavirus replication

The observation that HMGCR-dependent pathway was essential for rotavirus replication raised the question as to which downstream metabolite of the HMGCR-dependent/mevalonate pathway was necessary for rotavirus replication. To explore that, following the mevalonate pathway (Figure 2a), we next inhibited the pathway by a downstream inhibitor, 6-Fluoromevalonate, which targets mevalonate-pyrophosphate decarboxylase (MPD) by an ATP-dependent decarboxylation.^31^ The RNA copies of the intra- and extracellular rotavirus were markedly lower by 6-fluoromevalonate treatments in Caco2 cells, and the reductions were down to 40% and 35%, respectively, at the maximum 200 µM concentration, as well as the dramatic decreases on the rotavirus VP4 and VP6 proteins (Figure 4a, Figure S2a, Figure 5d). As evident from Figure 4b, g, and j, Figure S2a, Figure 5f and g, neither MA104 cells nor HSI organoids could sustain rotavirus replication in the presence of 200 µM 6-fluoromevalonate. The data indicated that 6-fluoromevalonate also exerted a great anti-rotavirus effect, suggesting the effective metabolite which influenced rotavirus replication could be some far downstream metabolite.

The article "Statins significantly repress rotavirus replication through downregulation of cholesterol synthesis" was retracted in 2022. Reasons: no approval from the institution; concerns about the authorship.

**Figure 4.** **The inhibitors of cholesterol biosynthesis impair rotavirus replication**. With rotavirus SA11 strain (MOI 0.7) infection and subsequently treated with different concentrations of 6-fluoromevalonate for 48 hours. The intra- and extracellular rotavirus RNA levels were measured by qRT-PCR (n = 6) (left) and the expressions of rotavirus VP4 protein were tested by western blot (right) in Caco2 cells (a), and in MA104 cells (b). With ZA-A treatments, the intra- and extracellular rotavirus RNA levels (n = 9) (left) and the expressions of rotavirus VP4 protein (right) in Caco2 cells (c), and in MA104 cells (d). with 1.25 µM U18666A treatment, the intra- and extracellular rotavirus RNA levels (n = 6) (left) and the expressions of rotavirus VP4 protein (right) in Caco2 cells (e), and in MA104 cells (f). In HSI organoids, the inner rotavirus RNA level with 200 µM 6-fluoromevalonate (n = 5) (g), 50 µM ZA-A (n = 5) (h) and 1.25 µM U18666A (n = 4) (i); and the expressions of rotavirus VP4 protein with 200 µM 6-fluoromevalonate or 50 µM ZA-A treatment (left) (j), with 1.25 µM U18666A treatment (right) (k). All data presented as mean ± SEM, *p < .05, **p < .01, ***p < .001

**Figure 5.** **The rotavirus titers and VP6 protein expressions of 200 µM 6-Fluoromevalonate, 50 µM ZA-A or 1.25 µM U18666A treatment**. The titers of infectious rotavirus particles were measured with 200 µM 6-Fluoromevalonate (a), 50 µM ZA-A (b) or 1.25 µM U18666A (c) treatment respectively (n = 6). Following the infection of rotavirus SA11 strain (MOI 0.7) with 200 µM 6-Fluoromevalonate or 50 µM ZA-A treatment respectively for 48 hours, the expression of rotavirus VP6 protein was observed in Caco2 cells (d), the expression of rotavirus VP6 protein was observed with 1.25 µM U18666A treatment in Caco2 cells (e), and the rotavirus VP6 expressions with the above treatments in MA104 cells (f) and HSI organoids (g). VP6 protein was green, and the nuclei of the cells were visualized by DAPI (blue). The results indicated that the inhibitors reduced the expressions of rotavirus VP6 protein

ZA-A targets Farnesyl-diphosphate farnesyltransferase 1 (FDFT1) which is a downstream enzyme blow MPD in the mevalonate pathway.^32^ qRT-PCR analysis showed that the intra- and extracellular rotavirus RNA copies apparently decreased (Figure 4c), and the expressions of VP4 and VP6 proteins also obviously reduced (Figure 4c, Figure S2b, Figure 5d). In MA104 cells, the intracellular and secreted rotavirus RNA copies decreased to 50% and 40%, respectively, by 50 µM ZA-A treatment (Figure 4d), and the VP4 and VP6 proteins also greatly decreased (Figure 4d, Fig. S2b, and Figure 5f). The anti-rotavirus effect of ZA-A also showed in the HSI organoids (Figure 4h and j, Figure S2b, Figure 5g). The data indicated that ZA-A also could downregulate rotavirus replication, implying some more far downstream metabolite might influence rotavirus replication.

The article "Statins significantly repress rotavirus replication through downregulation of cholesterol synthesis" was retracted in 2022. Reasons: no approval from the institution; concerns about the authorship.

U18666A is an inhibitor that targets desmosterol reductase and sterol–D8–D7 isomerase and oxidosqualene cyclase (OSC) in the mevalonate pathway to specifically block cholesterol production.^33^ By 1.25 µM U18666A treatment, the intra- and extracellular rotavirus RNA copies were summarized by qRT-PCR analysis in Caco2 cells (Figure 4e). U18666A dropped the intra- and extracellular virus RNA to around 40% similarly. Moreover, there were also significant decreases in the rotavirus VP4 and VP6 proteins (Figure 4e, Figure S2c, Figure 5e). In MA104 cells, U18666A showed the decreases to 26% and 38% of rotavirus RNA copies in the intra- and extracellular respectively, and the western blotting and IF staining results further confirmed that (Figure 4f, Figure S2c, Figure S5f). As shown in Figure 4i and k, Figure S2c, Figure 5g, U18666A suppressed rotavirus replication in HSI organoids. These results revealed that the decrease of cholesterol production repressed rotavirus replication.

Additionally, we also observed the harmful effects of 6-Fluoromevalonate, ZA-A, and U18666A on the titers of infectious rotavirus particles (Figure 5a, b, c). Taken together, these data indicated that cholesterol biosynthesis was connected with rotavirus replication. As shown in Figure S3a and b, the IC_50_ results of 6-Fluoromevalonate, ZA-A were far more than the maximal test concentrations, it indicated that their inhibitory effects on rotavirus replication were the cellular viability-independent. As shown in Figure S3c, no significant decrease in the cellular viability was observed with 1.25 µM U18666A treatment.

The article "Statins significantly repress rotavirus replication through downregulation of cholesterol synthesis" was retracted in 2022. Reasons: no approval from the institution; concerns about the authorship.

### Enhancement of cholesterol production upregulated rotavirus replication

We have verified that the inhibition of cholesterol synthesis suppressed rotavirus replication; theoretically, more cholesterol could enhance the virus replication. To address this question, we performed the experiment with R-MA that is a relevant enantiomer of mevalonate which is a critical substrate for cholesterol synthesis and direct cholesterol treatment, respectively, to observe the potential effects. A series concentrations of R-MA increased the intracellular and secreted rotavirus RNA copies in Caco2 cells, up to 2.5-fold and 3.2-fold respectively (Figure 6a). The increased expressions of the rotavirus VP4 and VP6 proteins were also obtained (Figure 6a, Figure S4a, Figure 7a). In MA014 cells, the results were similar (Figure 6b; Figure S4c, Figure 7b). In HSI organoids, 1,000 µM R-MA treatment resulted in 2.2-fold increase of the inner rotavirus RNA level, and the minor increases of the VP4 and VP6 proteins (Figure 6e, Figure S4e, Figure 7c). These results demonstrated that the enhancement of the mevalonate pathway increased rotavirus replication.

**Figure 6.** **Enhancement of cholesterol production provokes rotavirus replication**. With rotavirus SA11 strain (MOI 0.7) infection and subsequently treated with different concentrations of R-MA for 48 hours and subsequently the intra- and extracellular rotavirus RNA levels were measured by qRT-PCR (n = 5) (left) and the expressions of rotavirus VP4 protein were tested by western blot (right) in Caco2 cells (a), and in MA104 cells (b). With different concentrations of cholesterol treatment, the intra- and extracellular rotavirus levels (n = 5) (left) and the expressions of rotavirus VP4 protein (right) in Caco2 cells (c), and in MA104 cells (d). In HSI organoids, the inner rotavirus RNA level (n = 3) (left) and the expressions of rotavirus VP4 protein (right) with R-MA treatment (e), with cholesterol treatment (f). (g) The titers of infectious rotavirus particles were measured by TCID_50_ assay upon R-MA (n = 6) (left) or cholesterol (n = 6) (right) treatment respectively in MA104 cells. (h) The time-course experiment of 150 µM cholesterol treatment on the intracellular rotavirus replication. All data presented as mean ± SEM, *p < .05, **p < .01, ***p < .001

**Figure 7.** **Rotavirus VP6 expressions by R-MA or cholesterol treatment**. Rotavirus SA11 strain (MOI 0.7) infected Caco2 cells with 1,000 µM R-MA or 150 µM cholesterol treatment for 48 hours respectively in Caco2 cells (a), MA104 cells (b) and HSI organoids (c). Rotavirus VP6 protein was green, and the nuclei of the cells were visualized by DAPI (blue). The results showed that both of R-MA and cholesterol markedly increased the expressions of rotavirus VP6 protein

Next, we tested the effect of cholesterol on rotavirus infection. Respectively, we observed that there were 4.3-fold and 1.8-fold greater in the intra- and extracellular rotavirus RNA levels and the obvious increases of the rotavirus VP4 and VP6 proteins in Caco2 cells (Figure 6c, Figure S4b, Figure 7a). The semblable enhancements of rotavirus replication were also observed in MA104 cells (Figure 6d, Figure S4d, Figure 7d) and in HSI organoids (Figure 6f, Figure S4f, Figure 7c).

The article "Statins significantly repress rotavirus replication through downregulation of cholesterol synthesis" was retracted in 2022. Reasons: no approval from the institution; concerns about the authorship.

There were also the significant increases of rotavirus titer by 1,000 µM R-MA or 150 µM cholesterol treatment (Figure 6g). By a 96-h time course test, 150 µM cholesterol treatment gained a marked rise of the intracellular rotavirus RNA level (Figure 6h). All these results indicated that rotavirus replication could be upregulated by more cholesterol production. IC_50_ assays indicated that 1,000 µM R-MA or 150 µM cholesterol did not alter the viabilities of Caco2 and MA104 cells (Figure S4g and h).

## Combinations of HMGCR inhibition and cholesterol enhanced rotavirus replication

To further confirm the interaction between cholesterol metabolism and rotavirus replication, we measured the effects of the combinations of HMGCR inhibition by atorvastatin or shRNA HMGCR knockdown and cholesterol on rotavirus replication. Caco2 cells were infected with rotavirus SA11 strain and cultured by the combination of 50 µM atorvastatin and 150 µM cholesterol, and the combination of HMGCR knockdown Caco2 cells and 150 µM cholesterol. The levels of the intra- and extracellular rotavirus RNA by the combination of atorvastatin and cholesterol were more than the control, but less than the only cholesterol treatment (Figure 8a). We speculated that there was more cholesterol due to the contribution of the mevalonate pathway in the only cholesterol treatment group, which resulted in a higher rotavirus RNA level compared to the combination group. Consistent with the rotavirus RNA results, the combination treatment also increased the expressions of the rotavirus VP4 and VP6 proteins, but the increased extent was lower than the only cholesterol treatment (Figure 8b, Figure 9a, Figure 9d). In MA104 cells, the results were similar as these in Caco2 cells (Figure 8c and d, Figure 9d and e).

**Figure 8.** **Cholesterol provokes rotavirus replication in the absence of HMGCR activity**. With rotavirus SA11 strain (MOI 0.7) infection and subsequently treated with the combination of 50 µM atorvastatin and 150 µM cholesterol for 48 hours respectively. The intra- (left) and extracellular (right) rotavirus RNA levels were measured by qRT-PCR in Caco2 cells (n = 8) (a), and in MA104 cells (n = 6) (c). The expressions of rotavirus VP4 protein were measured by western blot in Caco2 cells (b), and in MA104 cells (d). With rotavirus SA11 infection (MOI 0.7), sh10952 and sh10955 HMGCR knockdown Caco2 cells were treated with 150 µM cholesterol for 48 hours. The intra- (left) and extracellular (right) rotavirus RNA levels (n = 4) (e) and the expression of rotavirus VP4 protein (f). All data presented as mean ± SEM, *p < .05, **p < .01, ***p < .001

**Figure 9.** **Rotavirus VP4 and VP6 proteins expressions of the combinations of atorvastatin or HMGCR knockdown and cholesterol treatment**. Western blot analysis of the expressions of rotavirus VP4 protein with the combinations of 50 µM atorvastatin and 150 µM cholesterol in Caco2 cells (n = 3) (a), MA104 cells (n = 3) (b), and with the combinations of HMGCR knockdown and 150 µM cholesterol (n = 3) (c). The visual aspects of the combinations of 50 µM atorvastatin and 150 µM cholesterol in Caco2 cells (d), and MA104 cells (e), and with the combinations of HMGCR knockdown and 150 µM cholesterol treatment (f). The results showed that the combinations of atorvastatin or HMGCR knockdown and cholesterol treatment significantly increased the rotavirus replications

With the combination of HMGCR knockdown and 150 µM cholesterol, rotavirus replication also significantly increased with exogenous cholesterol treatment in the HMGCR deficiency cells (Figure 8e and f, Figure 9c and f). Thus, these results suggested that cholesterol played a critical role in rotavirus replication.

The article "Statins significantly repress rotavirus replication through downregulation of cholesterol synthesis" was retracted in 2022. Reasons: no approval from the institution; concerns about the authorship.

### Cholesterol synthesis was a rate-limiting step for clinical rotavirus isolate replication

To avoid these results were rotavirus-specific strain-dependent, we tested the effects of all the compounds using a clinical rotavirus isolate, 026 K strain. Because the rotavirus 026 K RNA copies in supernatant were too low to be measured by qRT-PCR, only the intracellular rotavirus 026 K RNA copies were tested. There were the notable decreases to 24%, 17%, and 21% by atorvastatin, lovastatin and simvastatin treatments, respectively, compared to the control in the intracellular rotavirus 026 K RNA level (Figure 10a). The data indicated that the anti-rotavirus effects of the statins were rotavirus strain-independent, but the inhibitory effects might be distinct among different rotavirus strains. In the two HMGCR knockdown Caco2 cell lines, the rotavirus isolated replications were also significantly repressed (Figure 10b). Similar inhibitory effects also were observed by 6-fluoromevalonate, ZA-A and U18666A treatments, respectively (Figure 10c,d and e). R-MA and cholesterol significantly enhanced the rotavirus RNA productions to 1.7-fold and 10.6-fold, respectively (Figure 10f and g). The data indicated that the interaction between cholesterol and rotavirus was rotavirus strain-independent.

**Figure 10.** **Canonical cholesterol biosynthesis is the rate-limiting step for a rotavirus clinical isolate 026 K replication in Caco2 cells**. With the rotavirus 026 K strain infection, subsequently the intracellular rotavirus RNA levels were measured by qRT-PCR, after 48 hours treated with 50 µM atorvastatin (n = 4), or lovastatin (n = 4), or simvastatin (n = 6) treatment respectively (a), in sh10952 and sh10955 HMGCR knockdown Caco2 cells (b), with 6-fluoromevalonate treatment (n = 4) (c), with ZA-A treatment (n = 5) (d), with U18666A treatment (n = 6) (e), with R-MA treatment (n = 8) (f), with cholesterol treatment (n = 8) (g). All data presented as mean ± SEM, *p < .05, **p < .01, ***p < .001

## Discussion

The alteration of host cholesterol metabolism is a prominent feature in infections of multiple viruses, as these viruses need to modify host cholesterol homeostasis to fulfill the demands of their life cycles. West Nile virus (WNV) upregulates cholesterol synthesis to promote its replication; on the contrary, reducing cholesterol production by HMGCR inhibition had an inhibitory effect on WNV replication.^8^ Hepatitis C virus (HCV) infection leads to the activation of nuclear factor-κB (NF-κB) which can induce the expressions of heparan sulfate proteoglycans (HSPGs) for the upregulations of cholesterol uptake and HCV entry.^34^ Nevertheless, not all viruses adopts the strategy of increasing cholesterol metabolism. Kaposi’s sarcoma-associated herpesvirus (KSHV) encodes multiple miRNAs to target several enzymes of the mevalonate pathway to downregulate cholesterol synthesis, which promotes KSHV infection.^35^ Logically, host cells may take the opposite police on cholesterol homeostasis against viruses. Some HCV infected cells can downregulate the transcription of sterol regulatory element-binding protein 2 (SREBP2) which is a vital promoter for cholesterol production for repressing HCV replication. In clinical practice, the drugs which can inhibit cholesterol synthesis have shown the potentiality against HCV infection.^36^

The delicate interaction between the viruses and cholesterol provides a novel view for antivirus research, that inspires us to battle with the infections of several viruses through controlling cholesterol homeostasis. MβCD can suppress the infections of dengue virus and HCV.^37,38^ As a clinical drug, statin has pleiotropic effects to impair the replications of various viruses. Based on the cholesterol-lowering mechanism, statin can prevent influenza virus infection and minimize its severity,^39^ and exhibit anti-HCV activity,^40^ and also repress dengue virus replication.^41^ Besides, statin may perform the antiviral effects through its immunomodulatory function. It has been suggested that statin diminishes human immunodeficiency virus 1 (HIV-1) attachment to target cells by suppressing the interaction of intercellular adhesion molecule 1 (ICAM-1) and leukocyte function-associated antigen-1 (LFA-1).^42^

The article "Statins significantly repress rotavirus replication through downregulation of cholesterol synthesis" was retracted in 2022. Reasons: no approval from the institution; concerns about the authorship.

The conclusion of neither the interaction of cholesterol metabolism and rotavirus nor a clinical drug that is available to suppress rotavirus infection is available to date. According to the established links of cholesterol biosynthesis and the replications of multiple viruses, we explored the potential roles of different clinically used statins on rotavirus replication and clarified the relation between cholesterol metabolism and rotavirus replication. In our study, the tested three statins significantly inhibited rotavirus in all the pre-clinical models. The genetic knockdown of HMGCR mimicked the anti-rotavirus effect to exclude the pharmacological off-target effect of statin. Further, we used a variety of chemical inhibitors in the mevalonate pathway to confirm that cholesterol synthesis played an important role in rotavirus infection. By reverse verification, more cholesterol production upregulated rotavirus replication. The combination experiments proved the supportive function to rotavirus.

Nutrition management is the critical component of rotavirus infection care both during and after an episode of diarrhea.^43^ Despite few clinical studies are having reported the association between cholesterol diet and rotavirus-infected care, our research suggests that high cholesterol intake might support rotavirus infection, implying that the low cholesterol diet might be able to create an unfavorable environment for the virus replication. Note particularly both rotavirus infection/replication and cholesterol absorption occur in the mature enterocytes of the small intestine,^7,44^ which provides the theoretical possibility of their direct interaction. Unlike adults, as infants with the special physiological characteristic, dietary source contributes the majority of cholesterol pool,^45^ which highlights the potential significance of optimized nutrition strategy to moderate rotavirus infection in children. Due to the impact of rotavirus on the public health system, it is of interest to explore the modulation of nutritional compounds for the virus-infected patients.

The article "Statins significantly repress rotavirus replication through downregulation of cholesterol synthesis" was retracted in 2022. Reasons: no approval from the institution; concerns about the authorship.

Comparing to the small-molecule inhibitors, which have been developing and the pharmacology of antisense based nucleic acids in clinical trials, statin has the obvious advantages on safety. However, further studies regarding the efficacy in vivo and the pharmacokinetics of statin in children are essential to evaluate its potential as an antiviral drug. The molecular mechanism of how changes on cholesterol homeostasis affects rotavirus replication also requires more researches. Together, we hope that the study not only elaborates on the significance of cholesterol metabolism for rotavirus replication but also makes statin to emerge the potential preferred choice for controlling fulminant rotavirus-induced disease.

## Supplementary Material

Supplemental Material

## Data Availability

Raw data were generated at Erasmus MC. The data that support the findings of the study are available from the corresponding author, SD, upon reasonable request. Dataset availability is not applicable to this article as no new data were created or analyzed in the study.

## References

[1] VelazquezFR, MatsonDO, CalvaJJ, GuerreroL, MorrowAL, Carter-CampbellS, GlassRI, EstesMK, PickeringLK, Ruiz-PalaciosGM, et al. Rotavirus infection in infants as protection against subsequent infections. N Engl J Med. 1996;335(14):1022–19. doi:10.1056/NEJM199610033351404.8793926

[2] CrawfordSE, RamaniS, TateJE, ParasharUD, SvenssonL, HagbomM, FrancoMA, GreenbergHB, O’RyanM, KangG, et al. Rotavirus infection. Nat Rev Dis Primers. 2017;3(1):17083. doi:10.1038/nrdp.2017.83.29119972PMC5858916

[3] TateJE, BurtonAH, Boschi-PintoC, SteeleAD, DuqueJ, ParasharUD, et al. 2008 estimate of worldwide rotavirus-associated mortality in children younger than 5 years before the introduction of universal rotavirus vaccination programmes: a systematic review and meta-analysis. Lancet Infect Dis. 2012;12(2):136–141. doi:10.1016/S1473-3099(11)70253-5.22030330

[4] DesselbergerU.Differences of rotavirus vaccine effectiveness by country: likely causes and contributing factors. Pathogens. 2017. 6.10.3390/pathogens6040065PMC575058929231855

[5] ParkerEP, RamaniS, LopmanBA, ChurchJA, Iturriza-GomaraM, PrendergastAJ, GrasslyNC, et al. Causes of impaired oral vaccine efficacy in developing countries. Future Microbiol. 2018;13(1):97–118. doi:10.2217/fmb-2017-0128.29218997PMC7026772

[6] TelmesaniAM. Oral rehydration salts, zinc supplement and rota virus vaccine in the management of childhood acute diarrhea. J Family Community Med. 2010;17(2):79–82. doi:10.4103/1319-1683.71988.21359029PMC3045093

[7] LundgrenO, SvenssonL. Pathogenesis of rotavirus diarrhea. Microbes Infect. 2001;3(13):1145–1156. doi:10.1016/S1286-4579(01)01475-7.11709295PMC7128947

The article "Statins significantly repress rotavirus replication through downregulation of cholesterol synthesis" was retracted in 2022. Reasons: no approval from the institution; concerns about the authorship.

[8] MackenzieJM, KhromykhAA, PartonRG. Cholesterol manipulation by west Nile virus perturbs the cellular immune response. Cell Host Microbe. 2007;2(4):229–239. doi:10.1016/j.chom.2007.09.003.18005741

[9] AzzamKM, FesslerMB. Crosstalk between reverse cholesterol transport and innate immunity. Trends Endocrinol Metab. 2012;23(4):169–178. doi:10.1016/j.tem.2012.02.001.22406271PMC3338129

[10] Amini-Bavil-OlyaeeS, ChoiYJ, LeeJH, ShiM, HuangIC, FarzanM, JungJ, et al. The antiviral effector IFITM3 disrupts intracellular cholesterol homeostasis to block viral entry. Cell Host Microbe. 2013;13(4):452–464. doi:10.1016/j.chom.2013.03.006.23601107PMC3646482

[11] AriasCF, Silva-AyalaD, LopezS, TsaiB. Rotavirus entry: a deep journey into the cell with several exits. J Virol. 2015;89(2):890–893. doi:10.1128/JVI.01787-14.25378490PMC4300671

[12] SapinC, ColardO, DelmasO, TessierC, BretonM, EnoufV, ChwetzoffS, OuanichJ, CohenJ, WolfC, et al. Rafts promote assembly and atypical targeting of a nonenveloped virus, rotavirus, in Caco-2 cells. J Virol. 2002;76(9):4591–4602. doi:10.1128/JVI.76.9.4591-4602.2002.11932424PMC155075

[13] IsaP, RealpeM, RomeroP, LopezS, AriasCF. Rotavirus RRV associates with lipid membrane microdomains during cell entry. Virology. 2004;322(2):370–381. doi:10.1016/j.virol.2004.02.018.15110534

[14] GoldsteinJL, BrownMS. Regulation of the mevalonate pathway. Nature. 1990;343(6257):425–430. doi:10.1038/343425a0.1967820

[15] EndoA. The discovery and development of HMG-CoA reductase inhibitors. J Lipid Res. 1992;33(11):1569–1582. doi:10.1016/S0022-2275(20)41379-3.1464741

[16] RayKK, SRS, ErqouS, SeverP, JWJ, FordI, et al. Statins and all-cause mortality in high-risk primary prevention: a meta-analysis of 11 randomized controlled trials involving 65,229 participants. Arch Intern Med. 2010;170(12):1024–1031. doi:10.1001/archinternmed.2010.182.20585067

[17] ArmitageJ. The safety of statins in clinical practice. Lancet. 2007;370(9601):1781–1790. doi:10.1016/S0140-6736(07)60716-8.17559928

[18] LuirinkIK, WiegmanA, KustersDM, HofMH, GroothoffJW, de GrootE, KasteleinJJP, HuttenBA, et al. 20-year follow-up of statins in children with familial hypercholesterolemia. N Engl J Med. 2019;381(16):1547–1556. doi:10.1056/NEJMoa1816454.31618540

[19] KodachLL, JacobsRJ, VoorneveldPW, WildenbergME, VerspagetHW, van WezelT, MorreauH, HommesDW, PeppelenboschMP, van den BrinkGR, et al. Statins augment the chemosensitivity of colorectal cancer cells inducing epigenetic reprogramming and reducing colorectal cancer cell ‘stemness’ via the bone morphogenetic protein pathway. Gut. 2011;60(11):1544–1553. doi:10.1136/gut.2011.237495.21551187

The article "Statins significantly repress rotavirus replication through downregulation of cholesterol synthesis" was retracted in 2022. Reasons: no approval from the institution; concerns about the authorship.

[20] ChenS, DingS, YinY, XuL, LiP, Peppelenbosch MPMP, PanQ, WangW, et al. Suppression of pyrimidine biosynthesis by targeting DHODH enzyme robustly inhibits rotavirus replication. Antiviral Res. 2019;167:35–44. doi:10.1016/j.antiviral.2019.04.005.30974126

[21] YinY, BijveldsM, DangW, XuL, van der EijkAA, KnippingK, et al. Modeling rotavirus infection and antiviral therapy using primary intestinal organoids. Antiviral Res. 2015;123:120–131. doi:10.1016/j.antiviral.2015.09.010.26408355

[22] SaxenaK, BluttSE, EttayebiK, ZengXL, BroughmanJR, CrawfordSE, KarandikarUC, SastriNP, ConnerME, OpekunAR, et al. Human intestinal enteroids: a new model to study human rotavirus infection, host restriction, and pathophysiology. J Virol. 2016;90(1):43–56. doi:10.1128/JVI.01930-15.26446608PMC4702582

[23] SchmittgenTD, LivakKJ. Analyzing real-time PCR data by the comparative C(T) method. Nat Protoc. 2008;3(6):1101–1108. doi:10.1038/nprot.2008.73.18546601

[24] PanQ, de RuiterPE, von EijeKJ, SmitsR, KwekkeboomJ, TilanusHW, GoldsteinJL, BrownMS, et al. Disturbance of the microRNA pathway by commonly used lentiviral shRNA libraries limits the application for screening host factors involved in hepatitis C virus infection. FEBS Lett. 2011;585(7):1025–1030. doi:10.1016/j.febslet.2011.02.035.21376045

[25] ThakurAK, FezioWL. A computer program for estimating ld50 ld 50 and its confidence limits using modified behrens-reed-muench cumulant method. Drug Chem Toxicol. 1981;4(3):297–305. doi:10.3109/01480548109018136.7338208

[26] DelmasO, BretonM, SapinC, Le BivicA, ColardO, TrugnanG. Heterogeneity of Raft-type membrane microdomains associated with VP4, the rotavirus spike protein, in Caco-2 and MA 104 cells. J Virol. 2007;81(4):1610–1618. doi:10.1128/JVI.01433-06.17135322PMC1797590

[27] ChongPH, SeegerJD, FranklinC. Clinically relevant differences between the statins: implications for therapeutic selection. Am J Med. 2001;111(5):390–400. doi:10.1016/S0002-9343(01)00870-1.11583643

[28] EstesMK, GrahamDY, GerbaCP, SmithEM. Simian rotavirus SA11 replication in cell cultures. J Virol. 1979;31(3):810–815. doi:10.1128/jvi.31.3.810-815.1979.229253PMC353508

[29] LiM, Izpisua BelmonteJC. Organoids - preclinical models of human disease. N Engl J Med. 2019;380(6):569–579. doi:10.1056/NEJMra1806175.30726695

[30] SchirrisTJ, RenkemaGH, RitschelT, VoermansNC, BilosA, van EngelenBG, et al. Statin-induced myopathy is associated with mitochondrial complex iii inhibition. Cell Metab. 2015;22(3):399–407. doi:10.1016/j.cmet.2015.08.002.26331605

[31] VoynovaNE, FuZ, BattaileKP, HerdendorfTJ, KimJJ, MiziorkoHM. Human mevalonate diphosphate decarboxylase: characterization, investigation of the mevalonate diphosphate binding site, and crystal structure. Arch Biochem Biophys. 2008;480(1):58–67. doi:10.1016/j.abb.2008.08.024.18823933PMC2709241

The article "Statins significantly repress rotavirus replication through downregulation of cholesterol synthesis" was retracted in 2022. Reasons: no approval from the institution; concerns about the authorship.

[32] DoR, KissRS, GaudetD, EngertJC. Squalene synthase: a critical enzyme in the cholesterol biosynthesis pathway. Clin Genet. 2009;75(1):19–29. doi:10.1111/j.1399-0004.2008.01099.x.19054015

[33] TakanoT, EndohM, FukatsuH, SakuradaH, DokiT, HohdatsuT. The cholesterol transport inhibitor U18666A inhibits type I feline coronavirus infection. Antiviral Res. 2017;145:96–102. doi:10.1016/j.antiviral.2017.07.022.28780424PMC7113792

[34] ZhangF, SodroskiC, ChaH, LiQ, LiangTJ. Infection of hepatocytes with HCV increases cell surface levels of heparan sulfate proteoglycans, uptake of cholesterol and lipoprotein, and virus entry by up-regulating SMAD6 and SMAD7. Gastroenterology. 2017;152(1):257–70 e7. doi:10.1053/j.gastro.2016.09.033.27693511PMC5547743

[35] SerquinaAKP, KambachDM, SarkerO, ZiegelbauerJM. Viral microRNAs repress the cholesterol pathway, and 25-hydroxycholesterol inhibits infection. mBio. 2017. 8.10.1128/mBio.00576-17PMC551370928698273

[36] YeJ. Reliance of host cholesterol metabolic pathways for the life cycle of hepatitis C virus. PLoS Pathog. 2007;3(8):e108. doi:10.1371/journal.ppat.0030108.17784784PMC1959368

[37] CarroAC, DamonteEB. Requirement of cholesterol in the viral envelope for dengue virus infection. Virus Res. 2013;174(1–2):78–87. doi:10.1016/j.virusres.2013.03.005.23517753

[38] AizakiH, MorikawaK, FukasawaM, HaraH, InoueY, TaniH, SaitoK, NishijimaM, HanadaK, MatsuuraY, et al. Critical role of virion-associated cholesterol and sphingolipid in hepatitis C virus infection. J Virol. 2008;82(12):5715–5724. doi:10.1128/JVI.02530-07.18367533PMC2395132

[39] EpiscopioD, AminovS, BenjaminS, GermainG, DatanE, LandazuriJ, LockshinRA, ZakeriZ, et al. Atorvastatin restricts the ability of influenza virus to generate lipid droplets and severely suppresses the replication of the virus. FASEB J. 2019;33(8):9516–9525. doi:10.1096/fj.201900428RR.31125254PMC6662987

[40] IkedaM, AbeK, YamadaM, DansakoH, NakaK, KatoN. Different anti-HCV profiles of statins and their potential for combination therapy with interferon. Hepatology. 2006;44(1):117–125. doi:10.1002/hep.21232.16799963

[41] RothwellC, LebretonA, YoungNC, LimJY, LiuW, VasudevanS, et al. Cholesterol biosynthesis modulation regulates dengue viral replication. Virology. 2009;389:8–19.1941974510.1016/j.virol.2009.03.025

[42] GiguereJF, TremblayMJ. Statin compounds reduce human immunodeficiency virus type 1 replication by preventing the interaction between virion-associated host intercellular adhesion molecule 1 and its natural cell surface ligand LFA-1. J Virol. 2004;78(21):12062–12065. doi:10.1128/JVI.78.21.12062-12065.2004.15479847PMC523291

The article "Statins significantly repress rotavirus replication through downregulation of cholesterol synthesis" was retracted in 2022. Reasons: no approval from the institution; concerns about the authorship.

[43] TaylorCE, GreenoughWB3rd.Control of diarrheal diseases. Annu Rev Public Health. 1989;10(1):221–244. doi:10.1146/annurev.pu.10.050189.001253.2655632

[44] DawsonPA, RudelLL. Intestinal cholesterol absorption. Curr Opin Lipidol. 1999;10(4):315–320. doi:10.1097/00041433-199908000-00005.10482134

[45] KapourchaliFR, SurendiranG, GouletA, MoghadasianMH. The role of dietary cholesterol in lipoprotein metabolism and related metabolic abnormalities: a mini-review. Crit Rev Food Sci Nutr. 2016;56(14):2408–2415. doi:10.1080/10408398.2013.842887.26055276

